# Inception-LSTM Human Motion Recognition with Channel Attention Mechanism

**DOI:** 10.1155/2022/9173504

**Published:** 2022-06-13

**Authors:** Yongtao Xu, Liye Zhao

**Affiliations:** ^1^School of Instrument Science and Engineering, Southeast University, Nanjing 210096, China; ^2^Key Laboratory of Micro-Inertial Instrument and Advanced Navigation Technology, Ministry of Education, Southeast University, Nanjing 210096, China

## Abstract

An improved channel attention mechanism Inception-LSTM human motion recognition algorithm for inertial sensor signals is proposed to address the problems of high cost, many blind areas, and susceptibility to environmental effects in traditional video image-oriented human motion recognition algorithms. The proposed algorithm takes the inertial sensor signal as input, first extracts the spatial features of the sensor signal into the feature vector graph from multiple scales using the Inception parallel convolution structure, then uses the improved ECA (Efficient Channel Attention) channel attention module to extract the critical details of the feature vector graph of the sensor data, and finally uses the LSTM network to further extract the temporal features of the inertial sensor signals to achieve the classification and recognition of human motion posture. The experiment results demonstrate that 95.04% recognition accuracy on the public dataset PAMAP2 and 98.81% accuracy on the self-built dataset can be realized based on the algorithm model, indicating that the algorithm model has a superior recognition effect. In addition, the results of the visual analysis of channel attention weights show that the proposed model is interpretable for the recognition of human motions and is consistent with the living intuition.

## 1. Introduction

Lately, human motion recognition has turned into the most dynamic and famous area because of its wide application in true situations like medical care, smart home, and monitoring [1–3]. Traditional computer vision-based human motion recognition [4, 5] is limited in its effectiveness in the actual recognition process due to variations in illumination, complex background environments, and the influence of individual differences in objects. Compared with computer vision-based methods, inertial sensors have become increasingly important and started to be extensively applied in human motion recognition due to their low environmental coupling, high individual adaptability, and small size and low cost.

There are many existing studies on automatic human motion posture recognition based on inertial sensor data [6, 7], but accurate detection and recognition is still a challenge.The quality of the manually extracted signal features has a huge impact on the human motion recognition effect based on traditional machine learning algorithms (such as support vector machines [8] and random forests [9]), and thus, the professional knowledge in the field is required to transform sensor signal into corresponding feature expression for human motion recognition [10]. In addition, the elementary human postures can be represented effectually by the hand-made features, but they are unable to handle more complex motion patterns. In most cases, feature selection techniques are also needed to obtain significant features and reduce the dimension of feature space [11] to achieve optimal performance. To address these challenges, in-depth research on automatic feature extraction methods that do not require human intervention has become an active research area.

Convolutional neural networks (CNN) has emerged as a powerful tool in image processing and machine vision. When used for human action recognition of inertial sensors, convolutional neural networks can automatically extract high-dimensional data features and thus can largely avoid the reliance on feature engineering. Also, due to its rich expressive power and spatial feature extraction capability, it can achieve better results than traditional machine learning algorithms when processing inertial sensor data [12]. However, in existing studies, researchers have mostly used serial convolutional structures to deepen the depth of convolution [13, 14], while there are fewer studies on parallel convolutional structures to widen the convolution width for processing inertial sensor data. An Inception neural network structure was proposed in the literature [15]. This structure is established on convolutional neural network and adopts multipath parallel convolution mode, which improves the utilization rate of computing resources in the network and fully extracts spatial features of data on multiscale convolution kernel. It has excellent performance in the field of visual recognition and good scalability. LSTM is a special recurrent neural network (RNN) structure, which consists of a series of repeating neural networks combined in a chain. Its unique network structure makes it very sensitive to signals with temporal dependence. The attention mechanism is a widely studied network design approach in the fields of computer vision [16] and natural language processing [17]. Exhibiting a resemblance to human perception, the attention mechanism focuses upon the certain section of the objective region to magnify the key details of the object while abolishing other extraneous potentially baffling information, allowing neural network models to have a high level of interpretability. There are limited existing studies that apply attentional mechanisms to the field of inertial sensor action recognition. Literature [18] used a multihead model based on the SENet (Squeeze Excitation Network) channel attention mechanism to extract features from inertial sensors signal and attained good recognition results on the UCI and WISDM datasets. Literature [19] used a dual attention approach combining channel attention and spatial attention to achieve good action classification results on all four publicly available datasets. In literature [20], based on SENet, an optimized channel attention mechanism model ECA is proposed, which significantly reduces the complexity of the model through cross-channel interaction of feature information and the performance of the model has been raised simultaneously.

In order to deal with the problem that the human motion recognition algorithm based on video images is vulnerable to uncertainties in the environment in applications, and to overcome the limitation that traditional machine learning algorithms require expert knowledge in related fields for manual feature extraction, this paper proposes an Inception-LSTM human motion recognition algorithm that introduces a channel attention mechanism based on inertial sensor signals. The proposed human motion recognition algorithm automatically extracts spatial features of inertial sensor data using Inception convolutional structure, extracts temporal features of data using LSTM, and introduces an improved ECA channel attention mechanism module between the two feature extraction networks to make the model focus more on the critical details of sensor data features, suppress non-key information, and improve motion recognition rate.

## 2. Model Construction of the Inception-LSTM Algorithm for Introducing Channel Attention

The proposed Inception-LSTM human motion recognition algorithm, which introduces the channel attention mechanism, extracts the features of sensor signals in three parts: the spatial features of inertial sensor signals are extracted using a spatial feature extraction network; the model converges its attention on the key details of each action using a modified ECA channel attention module; and the temporal dependencies hidden in sensor signals are extracted using a temporal feature extraction network.

### 2.1. Spatial Feature Extraction Network

The multiaxial data output of acceleration and gyroscope of inertial sensors allows them to collect rich spatial features in characterizing human activities. And CNN have significant advantages in extracting spatial features of signals. Each feature pixel in the current neuron of a CNN is mapped to the previous layer of neurons by a local receptive field and then obtained by a nonlinear activation function. The calculation is shown in Equation (1).

(1) $$\begin{array}{c} s\left(i,j\right)=\sigma \left(\overset{H}{\underset{m=1}{\sum }}\overset{K}{\underset{n=1}{\sum }}w_{m,n}x_{i+m,j+n}+b\right), \end{array}$$

where *s*(*i*, *j*) is the feature pixel of the current neuron, *σ* is the nonlinear activation function, *w* is the weight matrix of the *H* × *K* convolution kernel, *b* is the bias, and *x* is the local receptive field of the upper layer neuron. CNN represent the data by convolution in order to abstract the features of the signals. Generally, the performance of convolutional neural network can be enhanced through increasing the depth and node number of each layer in serial sequential manner, but this brings two drawbacks: first, the larger network size makes the model risk of overfitting. Second, the amount of nodes in the network is too large, which makes the computational resources exponentially increase.

The Inception convolutional structure changes the serial sequential connection between layers of the traditional convolutional model by distributing four different convolutional kernels—one 1 × 1 convolution, one 1 × 1 convolution in series with a 3 × 3 convolution, one 1 × 1 convolution in series with a 5 × 5 convolution, and one 3 × 3 maximum pooling layer in series with a 1 × 1 convolution—on four different convolutional paths, and the input signals enter these 4 convolution paths in parallel in turn, and finally, the outputs of the 4 convolution results are stitched together and used as the input of the poststage network. This parallel convolution method can extract the spatial features of the input signal at different scales and give different weights to achieve a good recognition effect.

The proposed model in this paper adopts the Inception asymmetric convolution structure to construct a lightweight sensor signal space feature extraction module. As shown in Figure 1, from left to right, it is channel 1 to channel 4. Channel 1 performs two 1 × 1 convolution operations, similar to the fully connected operation in linear networks; channel 2 first performs a 1 × 1 convolution operation, aiming to trim the number of parameters and quicken the training process. Then, one 1 × 3 asymmetric convolution operation is performed to mine the feature information between acceleration and angular velocity of the inertial sensor and extract it into the feature vector graph through the convolution kernel of the lateral vector. Finally, a 3 × 1 convolution operation is performed to get the signal features in the same inertial axes of adjacent time into the feature vector map through the convolution kernel of longitudinal vectors; channel 3 first performs a 1 × 1 convolution operation with the same effect as in channel 2, then a 1 × 5 lateral convolution operation to expand the interaxis data features in a larger range into the feature map, and finally a 5 × 1 vertical convolution operation to fuse the temporal features of the data at a larger scale and add them to the feature map; channel 4 first introduces a maximum pooling layer to downsample the data samples composed of inertial sensor data to reduce the data dimensionality and compress the features and then performs a 1 × 1 convolution operation. The four channels of the altered Inception structure are independent of each other and process the data in parallel, and finally, the data of the four channels are stitched together by channel dimension. This asymmetric convolution structure can obtain the spatial features of inertial sensor signals better.

### 2.2. Channel Attention Mechanism

In the purpose of improving the performance of the proposed algorithm for inertial sensor signal recognition, the ECA channel attention mechanism module is introduced in this paper. ECA is an optimized channel attention mechanism model. Based on SENet, ECA can realize a huge complexity reduction and performance improvement of the model by a local cross channel interaction strategy without no reduction of the dimension and self-adaptive selection of 1D convolution kernel size. For a feature graph input *A* ∈ *R*^*W*×*H*×*C*^ with channel number *C*, height *H*, and width *W*, ECA first performs a global average pooling to compress the information of each channel independently to obtain a feature strip with dimension 1 × 1 × *C*. Then, the 1D convolution and nonlinear transformation are performed on the feature strip to obtain the attention weight *ω*_*i*_ for each channel *A*_*i*_. The weight *ω*_*i*_ for channel *A*_*i*_ focuses only on the current channel *A*_*i*_ and its *k* neighboring channels and is calculated as shown in Equation (2).

(2) $$\begin{array}{c} \omega_{i}=\sigma \left(\overset{k}{\underset{j=1}{\sum }}\omega_{i}^{j}A_{i}^{j}\right),A_{i}^{j}\in \Omega_{i}^{k}, \end{array}$$

where *Ω*_*i*_^*k*^ represents the set of *k* adjacent channels of *A*_*i*_^*j*^. The 1D convolution kernel size *k* is obtained by adaptive calculation of Equation (3), where *γ* = 2, *b* = 1.

(3) $$\begin{array}{c} k=\psi \left(C\right)=\left|\frac{\log_{2}\left(C\right)}{\gamma }+\frac{b}{\gamma }\right|. \end{array}$$

Based on the original ECA module, the proposed algorithm combines the inertial sensor signal to realize human motion recognition, and a channel feature extraction module is added in the later stage, as shown in Figure 2.

The algorithm put forward here is based on the original ECA module and combines the application context of human motion recognition with inertial sensor signals, adding a channel feature extraction module to its back-end, as shown in Figure 2.

The attention weights *ω*_*i*_ obtained from the original ECA module after the 1D convolution and nonlinear transformation are first arranged in descending order according to their absolute value magnitudes to obtain the sequence $\tilde{\omega }$ and its corresponding index. Then, the values of the first *N* sequences in sequence $\tilde{\omega }$ and their index values are selected. At the end of the multiplication of the original feature map input *A* ∈ *R*^*W*×*H*×*C*^ with the attention weights *ω*_*i*_, the corresponding feature channels of the multiplication results are extracted according to the indexes of the obtained values of the first *N* sequences, and the output feature map *A*′ ∈ *R*^*W*×*H*×*N*^ is finally obtained, where the parameter *N* is calculated by Equation (4).

(4) $$\begin{array}{c} N=k+{\left.\frac{\log_{2}\left(C\right)}{2}\right|}_{\text{even}}, \end{array}$$

where even indicates that the result is taken as the closest even number. By this extraction of the main feature channels, the feature utilization efficiency of the deep neural network is improved, which in turn improves the recognition performance of the network.

### 2.3. Temporal Feature Extraction Network

The signals generated by inertial sensors have strong temporal dependence when the human body performs various action posture activities, and RNN has significant advantages in extracting temporal features of the signals. The temporal features extracting network in the algorithm proposed in this paper consist of LSTM. Unlike RNN, LSTM introduces the concepts of input gate, forgetting gate, and output gate for realizing the update and output of memory states. Its basic neural network unit structure is shown in Figure 3.

In Figure 3, *c* is the cell state, which is similar to an information pipeline that runs through the entire operation cycle of the LSTM. The three gate structures of the LSTM allow for the removal and addition of information in the cell, allowing for selective information flow. *σ* is a nonlinear activation function that maps the output value of the function between 0 and 1, with 0 indicating no information passes and 1 indicating all information passes. *W* is the weight matrix, and *b* is the bias vector.

First, the forgetting gate determines what kind of message will be discarded from the cell. The gate will read the hidden state*h*_*t*−1_ of the prior moment with input *X*_*t*_ and output a value between [0,1] and the cell state *c*_*t*−1_ of the prior moment by the *σ* function to do the element multiplication operation. The result of the output*f*_*t*_ of the forgetting gate is illustrated in Equation (5).

(5) $$\begin{array}{c} f_{t}=\sigma \left(W_{f}\times \left[h_{t-1},X_{t}\right]+b_{f}\right). \end{array}$$

Second, the input gate determines what new messages are to be stored in the cell state The output of the *σ* function determines what values are to be updated and the tanh layer builds a new candidate cell state vector $\tilde{c_{t}}$ to determine in which way to add the output to the cell state. The output *i*_*t*_ of the input gate, the candidate cell state vector $\tilde{c_{t}}$, is updated with the current cell state *c*_*t*_as shown in Equation (6) to Equation (8).

(6) $$\begin{array}{c} i_{t}=\sigma \left(W_{i}\times \left[h_{t-1},X_{t}\right]+b_{i}\right), \end{array}$$

(7) $$\begin{array}{c} \tilde{c_{t}}=\tanh\left(W_{c}\times \left[h_{t-1},X_{t}\right]+b_{c}\right), \end{array}$$

(8) $$\begin{array}{c} c_{t}=f_{t}\times c_{t-1}+i_{t}\times \tilde{c_{t}}. \end{array}$$

Finally, the output of the LSTM is obtained from the output gate *o*_*t*_. The function *σ* determines which information will be output. The current cell state *c*_*t*_ is processed by tanh, and by the output of the *σ* function is multiplied by elements to obtain the final output *h*_*t*_ of the LSTM. The output *o*_*t*_ of the output gate and the final output *h*_*t*_ is illustrated according to Equation (9) to Equation (10).

(9) $$\begin{array}{c} o_{t}=\sigma \left(W_{o}\times \left[h_{t-1},X_{t}\right]+b_{o}\right), \end{array}$$

(10) $$\begin{array}{c} h_{t}=o_{t}\times \tanh\left(c_{t}\right). \end{array}$$

The design of the three gates in the LSTM makes the structure highly sensitive when dealing with data with temporal dependencies. For the temporal feature extraction module, its input at each time step is derived from the feature vector map extracted by the predecessor improved ECA module. At each time step, the LSTM reads in the feature map input *A*′ ∈ *R*^*W*×*H*×*N*^ line by line, and at time steps *t*_1_ to *t*_*n*_, a total of *n* data frames of the feature maps are read in. The LSTM network is used to take into account the interaction between the timing dimensions of the upstream and downstream inertial sensor data frames and to better extract the timing features.

In summary, the architecture of the proposed algorithm in this paper is presented in Figure 4.

## 3. Experimental Design

### 3.1. Experimental Data Acquisition

In the purpose of verifying the effectiveness of the proposed human motion recognition algorithm model, the recognition performance of the algorithm model is tested on the public dataset PAMAP2 and the self-built motion posture dataset, respectively.

The PAMAP2 human activity monitoring dataset [21] includes 18 different physical activity postures (e.g., cycling, running, and walking). The dataset was obtained from nine persons wearing three inertial measurement units, one at the wrist of the subject's dominant arm, one at the chest, and one at the ankle of the subject's dominant side of the body. According to the experimental requirements, each person was required to conduct 12 different activities, including sitting, standing, walking up and down stairs, jumping rope, and running. In addition, a number of random activities were performed for each program, including cleaning the room, driving, and working in front of the computer. Each inertial measurement unit was used with a sampling frequency of 100 Hz, and at each moment, three inertial measurement units collected acceleration, gyroscope, magnetometer, and body temperature data from the different body parts of the subject's current activity. A total of 216,000 data from 9 subjects were selected for the training. In the experiment, the dataset was split into training dataset and test dataset based on 7 : 3.

In the purpose of further verifying recognition capability and data robustness of the proposed model, a self-built human activity dataset was constructed in this paper. Two inertial measurement units are installed on the abdomen and the upper side of the knee of the left leg of the experimental tester, as shown in Figure 5. Each inertial measurement unit can output 3-axis gyroscope and 3-axis acceleration signal of the current activity of the tester. According to the experimental requirements, the tester needs to complete seven prescribed movements including sitting, standing, going upstairs, going downstairs, walking, running, and cycling. The long-time movements (sitting, standing, walking, running, and riding) are recorded as a set of data every 3 min, and the short-time movements (going upstairs and downstairs) are recorded as a set every 5 s. The sampling frequency of the inertial measurement unit was set to 25 Hz, and finally, 52,500 action data were obtained. During the training process, the dataset is also split into training dataset and test dataset based on 7 : 3.

### 3.2. Data Preprocessing

The preprocessing of the data is mainly for the processing of the missing values of the data and the segmentation of the data. For the missing values of the data, this paper mainly uses the method of Equation (11) for linear interpolation, where *y*_*i*_ is the missing value of the inertial sensor to be interpolated at the moment *x*_*i*_. *y*_*s*_ and *y*_*d*_ are the normal output sensor values at both ends of the missing value.

(11) $$\begin{array}{c} y_{i}=y_{s}+\frac{y_{d}-y_{s}}{x_{d}-x_{s}}\left(x_{i}-x_{s}\right). \end{array}$$

For data segmentation, an intelligent segmentation approach was used in literature [22] to adaptively adapt to human activity poses with different duration lengths, and good action recognition results were achieved under different conditions. However, the data segmentation method with fixed window size has obvious advantages in terms of computational efficiency, while it is easier to achieve end-to-end processing. Therefore, this paper uses the fixed-window-size strategy by referring to the approach in literature [23]. When the fixed window length is *K*, the data sequence for the same inertial measurement cell at the *i* window time is as follows:

(12) $$\begin{array}{c} \left\{\begin{array}{c} S_{i}^{a^{x}}=\left[a_{t}^{x},a_{t+1}^{x},\cdots ,a_{t+K-1}^{x}\right],\\ S_{i}^{a^{y}}=\left[a_{t}^{y},a_{t+1}^{y},\cdots ,a_{t+K-1}^{y}\right],\\ S_{i}^{a^{z}}=\left[a_{t}^{z},a_{t+1}^{z},\cdots ,a_{t+K-1}^{z}\right],\\ S_{i}^{g^{x}}=\left[g_{t}^{x},g_{t+1}^{x},\cdots ,g_{t+K-1}^{x}\right],\\ S_{i}^{g^{y}}=\left[g_{t}^{y},g_{t+1}^{y},\cdots ,g_{t+K-1}^{y}\right],\\ S_{i}^{g^{z}}=\left[g_{t}^{z},g_{t+1}^{z},\cdots ,g_{t+K-1}^{z}\right]. \end{array}\right. \end{array}$$

Different window lengths *K* will have an impact on the accuracy, and the relationship between several groups of window lengths *K* and accuracy is obtained by comparing the experiments as shown in Figure 6.

As can be seen from Figure 6, on the PAMAP2 dataset, the accuracy can reach about 95% when *K* is 100. On the self-built dataset, the accuracy can reach about 98% when *K* is 50. Therefore, the model training process sets *K* to 100 and 50 on the PAMAP2 dataset and the self-built dataset, respectively.

### 3.3. Model Training

The specific design parameters of the proposed Inception-LSTM human motion recognition algorithm that introduces the channel attention mechanism are shown in Table 1. The model is based on the Windows platform, running in the Anaconda environment of Python 3.6 kernel, and is obtained by CPU-accelerated training. During the training process, the hyperparameters learning rate and the number of training iteration are set to 0.001 and 200 respectively.

## 4. Experimental Results and Analysis

### 4.1. Evaluate Metrics

In this paper, the performance of the algorithm model is measured by using the evaluation metrics of average accuracy, precision, recall, and F1 value. The calculation formulas are Equation (13) to Equation (16), respectively.

(13) $$\begin{array}{c} \text{Accuracy}=\frac{\text{TP}+\text{TN}}{\text{TP}+\text{TN}+\text{FP}+\text{FN}}, \end{array}$$

(14) $$\begin{array}{c} \text{Precision}=\frac{\text{TP}}{\text{TP}+\text{FP}}, \end{array}$$

(15) $$\begin{array}{c} \text{Recall}=\frac{\text{TP}}{\text{TP}+\text{FN}}, \end{array}$$

(16) $$\begin{array}{c} \text{F}1=\frac{2\times \text{Precision}\times \text{Recall}}{\text{Precision}+\text{Recall}}, \end{array}$$

where TP means true positive, indicating a positive sample judged to be positive, TN means true negative, indicating a negative sample judged to be negative, FP means false positive, indicating a negative sample judged to be positive, and FN means false negative, indicating a positive sample judged to be negative.

### 4.2. Performance on the PAMAP2

In the purpose of observing the performance of the proposed algorithm on the public dataset PAMAP2, four algorithms, namely, the standard CNN network, the LSTM network, the neural network without channel attention mechanism, and the neural network with the original ECA added in the proposed model, are also designed as the control experiment of the proposed algorithm model in this paper. Meanwhile, in the purpose of ensuring the fairness of the comparison experiment, the parameters of the convolutional layers of the standard CNN network are set to the serial sequential connection form of the parameters of the Inception convolutional structure in this model to ensure the consistent scale of the convolutional layers. The parameters of the rest of the neural network algorithms are set with the same values of the proposed model. All adjustable hyperparameters were kept consistent with the proposed model during the experiments. The results are displayed in Figure 7.

As is displayed in Figure 7, the neural network without ECA that combines the Inception parallel convolutional structure with LSTM has significantly higher recognition accuracy than the classical CNN with serial sequential connections and the LSTM neural network alone. Meanwhile, the model incorporating the channel attention mechanism performs significantly better than the ordinary neural network without the channel attention mechanism in terms of recognition accuracy. In addition, the improved ECA model with channel feature extraction proposed in this paper also has a certain improvement in action recognition accuracy compared with the unimproved original ECA.

The proposed algorithm in this paper is compared with other algorithms in existing studies using the same PAMAP2 dataset, and the comparison results are displayed in Table 2. As is seen in the table, the proposed Inception-LSTM human action recognition algorithm that introduces a channel attention mechanism improves 1.88% in recognition accuracy compared to the literature [19] that uses a dual attention mechanism and improves over the AttnSense model proposed in the literature [24] and the layered convolutional neural network model with local loss proposed in the literature [25] by 5.74% and 2.07%. Also, the increase in model size is almost negligible compared to the neural network without the use of ECA.

The confusion matrix of the algorithm proposed in this paper is displayed in Figure 8. From the figure, it can be observed that the recognition accuracy of the algorithm can reach more than 90% for most of the actions on the PAMAP2 dataset. Among them, the recognition accuracy of rope jumping and running actions can reach 100%. For some more confusing actions such as sitting, standing, and ironing, the recognition effect is poor. Sitting actions are easily misclassified as standing actions and standing actions are easily misclassified as ironing. The demarcation between such static actions is not obvious, so they are often misclassified by the model.

In order to visualize the model interpretability brought by the channel attention mechanism, this paper provides a visual analysis of channel attention weights to evaluate the influence of various body parts on motion recognition when the human body performs different motion postures, and the results are displayed in Figure 9.

In Figure 9, the shades of the sensor colors at different moments indicate how much attention the algorithm model pays to the current activity on that component of the sensor. From the figure, it can be observed that the model proposed in this paper pays more attention to the *x*-axis component of the wrist sensor, the *x*-axis component of the chest sensor, and the *z*-axis component of the ankle sensor during the running activity. During the cycling activity, the model pays much attention to the *x*-axis and *z*-axis components of the ankle sensors. For the rope-jumping activity, the proposed model pays more attention to the *y*-axis and *z*-axis components of the wrist and the three axial components of the ankle. During the ironing activity, the model pays more attention to the *x*-axis and *y*-axis components at the wrist. Thus, it can be observed that the algorithm incorporating the channel attention mechanism is interpretable in terms of action recognition results and is generally consistent with the life intuition.

### 4.3. Performance on the Self-Built Dataset

The same four neural network algorithms, standard CNN network, LSTM network, neural network without channel attention mechanism, and the proposed model with original ECA neural network, were designed as control experiments on the self-built dataset. The adjustable hyperparameters of the models and the scale of the models are kept consistent with the proposed model. The experimental results are displayed in Figure 10.

As it can be observed from Figure 10, the proposed model has some improvement in accuracy over the model using the original ECA. Meanwhile, the neural network incorporating the channel attention mechanism is overall more accurate and converges faster than the neural network without the channel attention mechanism. The experimental results and model sizes of the different models on the self-built dataset are presented in Table 3.

The confusion matrix for the proposed model to identify each action in the self-built dataset is displayed in Figure 11.

As can be observed from Figure 11, the proposed model can maintain high accuracy in recognizing all seven motions on the self-built dataset. Among them, the recognition accuracy of sitting still, running, and cycling reaches 100%. Among them, the motion patterns of going upstairs, going downstairs, and walking are more similar, so the degree of confusion is higher.

The visualization results of the attention weights of the model are shown in Figure 12. As is shown in the figure, under the condition that the two inertial measurement units characterize the human activity posture, the channel attention model pays high attention to the signal component of the abdominal sensor *x*-axis when the human body is in the standing posture. During the upstairs activity, the channel attention model pays more attention to the signal components of the *x*-axis and *z*-axis of the leg sensors, which is consistent with the intuition of daily life.

## 5. Summary

In this paper, we propose the Inception-LSTM human motion recognition algorithm with the introduction of channel attention mechanism, which has two main features. One is to replace the traditional serial sequentially connected convolutional neural network with the Inception parallel convolutional structure to fully extract the spatial features of inertial sensors on multiple paths and scales and to join the LSTM network to extract the temporal features of the signals. Second, the channel attention mechanism ECA module is improved and fused into the neural network model by combining the inertial sensor signal characteristics to improve the recognition efficiency and resource utilization of the model. The proposed algorithm is tested on the public dataset PAMAP2 and the self-built dataset, and good recognition results are achieved on both datasets. The accuracy of the proposed algorithm for human motion recognition is higher than that of standard CNN, LSTM, and neural network models without using attention mechanism. Also, the improved ECA module has improved the recognition results compared with the original ECA module. In addition, the visual analysis of channel attention weights for several typical actions shows that the action recognition results of the proposed algorithm model are interpretable and consistent with the living intuition.

## Figures and Tables

**Figure 1:** Inception asymmetric convolution structure.

**Figure 2:** Improved ECA module structure.

**Figure 3:** Internal structure of LSTM.

**Figure 4:** Inception-LSTM algorithm model with channel attention.

**Figure 5:** Schematic diagram of the sensor wearing.

**Figure 6:** Influence of different window lengths on accuracy.

**Figure 7:** Accuracy of each model on PAMAP2 dataset.

**Figure 8:** The confusion matrix of different motions of the proposed model on PAMAP2 dataset.

**Figure 9:** Visualization of channel attention weights of different motions on PAMAP2 dataset.

**Figure 10:** Accuracy of each model on self-built dataset.

**Figure 11:** The confusion matrix of different motions of the proposed model on self-built dataset.

**Figure 12:** Visualization of channel attention weights of different motions on self-built dataset.

**Table 1:** The parameters of each layer of the proposed model.

Order number	Layer position	Size	Number of parameters
1	The convolutional layer, 1_1	[64, 1, 1, 1]	128
2	The convolutional layer, 1_2	[64, 64, 1, 1]	4160
3	The convolutional layer, 2_1	[64, 1, 1, 1]	128
4	Convolutional layer 2_21	[128, 64, 1, 3]	24704
5	Convolutional layer 2_22	[128, 128, 3, 1]	49280
6	The convolutional layer, 3_1	[64, 1, 1, 1]	128
7	Convolutional layer: 3_21	[128, 64, 1, 5]	41088
8	Convolutional layer 3_22	[128, 128, 5, 1]	82048
9	Maximum pooling layer	[64, 1, 3, 3]	0
10	Convolutional layer 4	[64, 1, 1, 1]	4160
11	Channel attention block	[1, 5]	385
12	Feature extraction layer	[9, 384, 1, 1]	3465
13	LSTM layer	[64, 18]	5312
14	Fully connected layer	[12, 64]	780

**Table 2:** Experimental results of different models on PAMAP2.

Algorithm model	Accuracy	Precision	Recall	F1 value	Model size
Classics CNN	91.11%	91.41%	91.11%	91.26%	7.14 M
LSTM	89.28%	89.69%	89.28%	89.49%	0.37 M
Neural network without ECA	92.44%	92.93%	92.44%	92.68%	2.67 M
Original ECA	93.91%	94.04%	93.91%	93.97%	2.68 M
This article model	95.04%	95.06%	95.21%	95.13%	2.68 M
Literature: [24]	89.30%	—	—	—	—
Literature: [25]	92.97%	—	—	—	—
Literature: [19]	93.16%	—	—	—	3.51 M

**Table 3:** Experimental results of different models on self-built dataset.

Algorithm model	Accuracy	Precision	Recall	F1 value	Model size
Classics CNN	95.71%	96.12%	95.71%	95.91%	2.53 M
LSTM	95.02%	95.98%	95.02%	95.50%	0.34 M
Neural network without ECA	96.77%	96.85%	96.77%	96.81%	1.21 M
Original ECA	98.44%	98.54%	98.44%	98.49%	1.24 M
The proposed model	98.81%	98.81%	98.81%	98.81%	1.24 M

## Data Availability

The datasets used during the current study are available from the corresponding author on reasonable request.
